# Trends in hepatitis B virus screening at the onset of chemotherapy in a large US cancer center

**DOI:** 10.1186/1471-2407-13-534

**Published:** 2013-11-09

**Authors:** Jessica P Hwang, Michael J Fisch, Anna S-F Lok, Hong Zhang, John M Vierling, Maria E Suarez-Almazor

**Affiliations:** 1 Department of General Internal Medicine, The University of Texas MD Anderson Cancer Center, 1515 Holcombe Blvd., Unit 1465, Houston, Texas 77030, USA; 2 University of Michigan, Ann Arbor, Michigan, USA; 3 Baylor College of Medicine, Houston, Texas, USA; 4 Department of General Oncology, The University of Texas MD Anderson Cancer Center, Houston, Texas, USA

**Keywords:** Hepatitis B virus, Hepatitis B virus screening, Chemotherapy, Reactivation

## Abstract

**Background:**

National organizations recommend screening for hepatitis B virus (HBV) before chemotherapy but differ regarding which patients should be screened. We aimed to determine contemporary screening rates at a cancer center and the possible influence on these rates of publication of national recommendations.

**Methods:**

We conducted a retrospective cohort study of HBV screening in cancer patients registered during the period from January 2004 through April 2011. Screening was defined as HBsAg and anti-HBc tests ordered around the time of initial chemotherapy. We compared screening rates for 3 periods: January 1, 2004, through December 18, 2008 (Food and Drug Administration and American Association for the Study of Liver Diseases 2007 recommendations); December 19, 2008, through September 30, 2010 (Centers for Disease Control and Prevention, National Comprehensive Cancer Network, American Association for the Study of Liver Diseases 2009, Institute of Medicine, and American Society of Clinical Oncology recommendations); and October 1, 2010, through April 30, 2011. Logistic regression models were used to identify predictors of screening.

**Results:**

Of 141,877 new patients, 18,688 received chemotherapy, and 3020 (16.2%) were screened. HBV screening rates increased over the 3 time periods (14.8%, 18.2%, 19.9%; *P* < 0.0001), but <19% of patients with HBV risk factors were screened. Among patients with hematologic malignancies, over 66% were screened, and odds of screening nearly doubled after publication of the recommendations (*P* < 0.0001). Less than 4% of patients with solid tumors were screened, although odds of screening increased 70% after publication of the recommendations (*P* = 0.003). Other predictors of screening included younger age, planned rituximab therapy, and known risk factors for HBV infection.

**Conclusions:**

Most patients with solid tumors or HBV risk factors remained unscreened, although screening rates increased after publication of national recommendations. Efforts are needed to increase awareness of the importance of HBV screening before chemotherapy to identify patients who should start antiviral prophylaxis.

## Background

National [1-7] and international [8,9] recommendations for hepatitis B virus (HBV) screening before chemotherapy emphasize the need to identify patients with HBV infection so that antiviral prophylaxis can be initiated to prevent reactivation of HBV infection. The pooled (range) incidence of HBV reactivation, HBV-related hepatitis, HBV-related liver failure, and HBV-related death among cancer patients receiving chemotherapy, who had not received antiviral prophylaxis has been reported to be 37% (24-88%), 33% (24-88%), 13% (5-33%) and 7% (0-63%), respectively [10]. The 7 national recommendations, however, differ regarding which patients should be screened [1-7] (Table 1). Unfortunately, no population-based studies have been conducted in the US to inform an evidence-based HBV screening policy.

**Table 1:** National recommendations

**Recommendation**	**Online publication date**	**Print publication date**	**Recommended screening practice**
^1^FDA Dear Healthcare Professional Letter	7/12/2004	Online only	Screen patients at high risk of HBV infection before initiation of rituximab therapy. Closely monitor carriers of HBV for clinical and laboratory signs of active HBV infection and for signs of hepatitis during and for up to several months after rituximab therapy.
^2^AASLD	1/26/2007	2/2007	Screen patients at high risk for HBV infection prior to immunosuppressive therapy.
			Test with HBsAg.
^3^CDC	9/19/2008	9/19/2008	Screen all patients prior to immunosuppressive therapies.
			Test with HBsAg, anti-HBc, and anti-HBs.
^4^AASLD Update	7/28/2009	9/2009	Screen patients at high risk for HBV infection prior to immunosuppressive therapy.
			Test with HBsAg and anti-HBc.
^5^NCCN	8/28/2009	Online only	Screen cancer patients with lymphoid malignancies, patients who have spent significant time in HBV-endemic areas or have risk factors for HBV infection, and patients anticipating intensive immunosuppressive therapy.
			Test with HBsAg, anti-HBc, and anti-HBs.
^6^IOM	1/11/2010	1/11/2010	Screen patients with HBV risk factors.
			Test with HBsAg.
^7^ASCO	6/1/2010	7/1/2010	Screen cancer patients at high risk for HBV infection or anticipating highly immunosuppressive therapy such as stem cell transplantation or rituximab therapy.
			Test with HBsAg and in some cases also with anti-HBc.

*Abbreviations*: *AASLD* American Association for the Study of Liver Diseases, *ASCO* American Society of Clinical Oncology, *CDC* Centers for Disease Control and Prevention, *FDA* Food and Drug Administration, *IOM* Institute of Medicine, *NCCN* National Comprehensive Cancer Network, *HBsAg* Hepatitis B surface antigen, *anti-HBc* Antibody to hepatitis B core antibody, *anti-HBs* Antibody to hepatitis B surface antigen.

Although the rates of HBV screening before immunosuppressive therapy in the US are unknown because of the lack of large-scale studies, rates have been estimated through physician surveys, which have shown rates ranging from 38-80% [11-13]. However, these studies were limited by the potential for recall bias and low survey response rates (5-63%). Furthermore, screening practices reported in these studies may not reflect actual screening practices.

We previously found that only 17% of patients treated at a US cancer center from 2004 through 2007 were screened for HBV infection before chemotherapy [14]. The purpose of this study was to update our previous study by determining HBV screening rates at the same cancer center from 2004 through 2011 and to examine the possible influence of national recommendations published between 2004 and 2010 on HBV screening rates over time.

## Methods

### Data sources

We conducted a retrospective cohort study of adults with newly diagnosed cancer who registered at The University of Texas MD Anderson Cancer Center between January 1, 2004, and April 30, 2011, and received chemotherapy. This study was approved by the MD Anderson Institutional Review Board. We merged patient data from 4 institutional sources:

1. Tumor Registry: patient demographics, including birthplace, and cancer type (hematologic malignancies vs. solid tumors); primary liver cancer was excluded because of the etiologic relationship between HBV and hepatocellular carcinoma. At MD Anderson, patient’s race/ethnicity can be ascertained based on self-reporting, reporting by the referring clinic, or assignment by administrative staff. We categorized race/ethnicity as White, Black, Hispanic, Asian, or Other. Birthplace in a region of moderate to high prevalence of HBV infection was considered a risk factor for HBV infection [3].

2. Pharmacy Informatics: chemotherapy drugs and dates administered. Chemotherapy was classified according to American Cancer Society classification [15]. We excluded oral chemotherapy because we could not validate medication dispensing dates. We excluded patients in therapeutic clinical trials since some clinical trials excluded patients with liver disease or hepatitis and screening for HBV was often dictated by the protocol and not reflective of the investigators’ decision.

3. Patient Accounts: ICD-9 codes corresponding to risk factors for HBV infection (see Table 2) anytime before the end of the screening period (defined below).

4. Laboratory Informatics: test dates and results for hepatitis B surface antigen (HBsAg), antibody to hepatitis B core antibody (anti-HBc), alanine aminotransferase, total bilirubin, and HBV DNA.

**Table 2:** Characteristics of the study population by screening status

	**All patients**	**Screened patients**	**Unscreened patients**	***P value***
	**(N = 18,688)**	**(N = 3020)**	**(N = 15668)**	
**Characteristic**	**No. (%)**^**a**^	**No. (%)**^**b**^	**No. (%)**^**b**^	
Age, years, mean (SD)	55.0 (13.5)	52.5 (15.4)	55.5 (13.0)	<0.0001
Sex				<0.0001
Female	10,608 (56.8)	1305 (12.3)	9303 (87.7)	
Male	8080 (43.2)	1715 (21.2)	6365 (78.8)	
Race/ethnicity				<0.0001
White	13,168 (70.5)	2168 (16.5)	11000 (83.5)	
Hispanic	2319 (12.5)	402 (17.3)	1917 (82.7)	
Black	2092 (11.2)	247 (11.8)	1845 (88.2)	
Asian	508 (2.7)	76 (15.0)	432 (85.0)	
Other	601 (3.2)	127 (21.1)	474 (78.9)	
US residence	18,090 (96.8)	2896 (16.0)	15194 (84.0)	0.002
HBV risk factor^c,d^	5391 (28.8)	1016 (18.8)	4375 (81.2)	<0.0001
Birthplace	1286 (6.9)	220 (17.1)	1066 (82.9)	
Abnormal liver function	368 (2.0)	170 (46.2)	198 (53.8)	
Hepatitis (not specified)	173 (0.9)	90 (52.0)	83 (48.0)	
Hepatitis C	213 (1.1)	104 (48.8)	109 (51.2)	
Other liver conditions	3821 (20.4)	610 (16.0)	3211 (84.0)	
HIV	70 (0.4)	39 (55.7)	31 (44.3)	
Drug abuse	39 (0.2)	15 (38.5)	24 (61.5)	
Sexually transmitted disease	106 (0.6)	36 (34.0)	70 (66.0)	
History of HBV infection^e^	78 (0.4)	20 (25.6)	58 (74.4)	0.02
Cancer type				<0.0001
Solid tumor^f^	15,031 (80.4)	581 (3.9)	14450 (96.1)	
Hematologic malignancy	3657 (19.6)	2439 (66.7)	1218 (33.3)	
Chemotherapy type				<0.0001
Rituximab	1977 (10.6)	1360 (68.8)	617 (31.2)	
Non-rituximab	16,711 (89.4)	1660 (9.9)	15051 (90.1)	

*Abbreviations*: *HBV* hepatitis B virus, *HIV* human immunodeficiency virus, *SD* standard deviation, *US* United States.

^a^The percentages represent column percentages (denominator equal to total number of patients in the study, 18,688). For example, 56.8% (10,608/18,688) of the patients in the study were women.

^b^The percentages represent row percentages (denominator equal to total number of patients with the given characteristic). For example, 12.3% (1305/10,608) of the females were screened for HBV infection while 87.7% (9303/10,608) were not.

^c^Patients born in countries with moderate to high prevalence of HBV infection according to the Centers for Disease Control and Prevention^3^ or at least 1 of the following ICD-9 diagnosis codes any time before chemotherapy were considered to have a risk factor for HBV infection:

(i) abnormal liver function (codes 794.8);

(ii) hepatitis, not specific (codes 070, 070.4, 070.49, 070.5, 070.59, 070.6, 070.9, 571.4, 571.40, 571.41, 571.42, 571.49, 573.1, 573.2, 573.3, v02.6, v02.60, and v02.69);

(iii) other liver conditions (codes 571, 571.0, 571.2, 571.3, 571.5, 571.6, 571.8, 571.9, 572, 572.0, 572.2, 572.8, 573, 573.8, 573.9, 782.4, 789.1, and 794.8);

(iv) hepatitis C (codes 070.41, 070.44, 070.51, 070.54, 070.7, 070.70, 070.71, and v02.62);

(v) HIV (codes 042, 042.0, 042.1, 042.2, 043, 043.0, 043.1, 043.2, 043.3, 044.0, 044.9, 079.53, 795.71, 795.8, v08, and v65.44);

(vi) drug abuse (codes 305.9, 305.90, 305.91, 305.92, 305.93);

(vii) sexually transmitted disease (codes 054.1, 054.10, 054.19, 078, 078.10, 078.11, 078.19, 078.8, 078.88, 079.8, 079.88, 079.9, 079.98, 091, 091.0, 091.1, 091.2, 091.3, 091.4, 091.5, 091.6, 091.69, 091.7, 091.8, 091.89, 091.9, 092, 092.0, 092.9, 093, 093.8, 093.89, 093.9, 094, 094.3, 094.8, 094.89, 094.9, 095, 095.1, 095.3, 095.4, 095.5, 095.6, 095.7, 095.8, 095.9, 096, 097, 097.0, 097.1, 097.9, 099.41, 099.50, 099.51, 099.52, 099.53, 099.54, 099.55, 099.56, 099.59, 483.1, v02.7, v73.8).

^d^Sum of patient numbers in the individual risk factor categories exceeds total number of patients with risk factors (n = 5391) since some patients had more than 1 HBV risk factor.

^e^We considered patients to have a history of HBV infection if they had an ICD-9 code for HBV infection (0.70.22, 0.70.23, 0.70.30, 0.70.32, 0.70.33, 0.70.44, 0.70.51, 0.70.54, 0.70.70, v02.61, v02.62) either 1) before HBV screening test among patients who were screened, or 2) before the second chemotherapy administration among patients who did not have HBV screening.

^f^Excludes primary liver cancer.

### HBV screening and infection

Screening was defined as having both HBsAg and anti-HBc tests ordered in the period from 2 months before the first administration of chemotherapy until the second administration of chemotherapy. MD Anderson has no official policy recommending prechemotherapy HBV screening. Positive findings on both HBsAg and anti-HBc tests were considered to indicate chronic HBV infection. Negative HBsAg test but positive anti-HBc test were considered to indicate occult HBV infection or convalescence after previous infection. Unfortunately, antibody to hepatitis B surface antigen (anti-HBs) test, which is positive in convalescence and negative in occult disease, was ordered in only 1% of patients.

### Three time periods

We used dates of the publication of national HBV recommendations to create 3 time intervals and categorized patients in these intervals according to date of first chemotherapy administration. We used 90 days after publication of recommendations as cut-off dates to allow adequate time for dissemination and potential change in practice patterns.

•Period 1: January 1, 2004, through December 18, 2008 (includes publication of Food and Drug Administration [FDA] letter [1] and 2007 American Association for the Study of Liver Diseases [AASLD] [2] recommendation).

•Period 2: December 19, 2008, through September 30, 2010 (includes publication of Centers for Disease Control and Prevention [CDC], [3] 2009 AASLD, [4] National Comprehensive Cancer Network [NCCN], [5] Institute of Medicine [IOM] [6] recommendations, and American Society of Clinical Oncology [ASCO] provisional clinical opinion [PCO] [7]).

•Period 3: October 1, 2010, through April 30, 2011 (after publication of above recommendations).

### Statistical methods

We calculated screening prevalence for each time period and tested for an increase in screening across the 3 periods using Cochran-Armitage trend tests. We compared characteristics of screened and unscreened patients using Pearson’s chi-square tests for categorical variables and Student’s *t*-test for continuous variables. We calculated screening rate per quarter and determined the rate of change of screening prevalence per quarter by cancer type and time period using regression analysis. Our main outcome variable was screening using HBsAg and anti-HBc tests. Independent variables included age, gender, race/ethnicity, US residency, having an HBV risk factor, cancer type, rituximab therapy, and date of first chemotherapy administration. We used 2 logistic regression models to identify predictors of screening, one for patients with solid tumors and one for patients with hematologic malignancies. We used backward elimination to select final models with a criterion of *P* > 0.05 for exclusion. Hosmer and Lemeshow goodness-of-fit tests were used to evaluate model fit. We determined the proportion of positive test results among screened patients and compared the rates of either a positive HBsAg test or a positive anti-HBc test result across the 3 time periods using Pearson’s chi-square test. We used SAS software, version 9.2 (SAS Institute, Cary, North Carolina), for statistical analyses.

## Results

During the study period, 141,877 new patients were registered at MD Anderson (Figure 1), of whom 18,688 (13.2%) received chemotherapy at MD Anderson. Overall, 3020 (16.2%) of the patients who received chemotherapy were screened for HBV infection around the onset of chemotherapy.

**Figure 1:** **Study patient population.** Flow diagram for study patients showing the exclusion of patients who did not have chemotherapy, had investigational chemotherapy, or non-parenteral routes of chemotherapy. Patients with primary liver cancer were also excluded.

The prevalence of HBV screening was approximately 4% (581/15,031) among patients with solid tumors and nearly 67% (2439/3657) among patients with hematologic malignancies. Nearly 29% (5391) of all patients had a risk factor for HBV infection, and less than 19% of these patients (1016) were screened. Over 10% (1977) of all patients received rituximab, and nearly 69% of these patients (1360) were screened. About 15% of the Asian patients and 12% of the Black patients were screened compared to nearly 17% of the White patients (Table 2).

The prevalence of HBV screening increased slightly across the 3 time periods, from 14.8% in period 1 to 18.2% in period 2 and 19.9% in period 3 (*P* < 0.001) (Table 3). For patients with known risk factors for HBV infection, screening prevalence increased over the 3 periods. For patients who received rituximab, screening prevalence increased between periods 1 and 2 and then decreased slightly in period 3. For Asian patients, screening prevalence did not change significantly over the 3 periods; for Black patients, screening prevalence increased over the 3 periods (Table 3).

**Table 3:** **Rates of HBV screening**^**a **^**by screening period**

**Characteristic**	**Period 1**^**b**^		**Period 2**^**c**^		**Period 3**^**d**^		***P *** **value**^**e**^
	**All patients**	**Screened patients**	**All patients**	**Screened patients**	**All patients**	**Screened patients**	
	**(N = 11,833)**	**(N = 1754)**	**(N = 5703)**	**(N = 1037)**	**(N = 1152)**	**(N = 229)**	
Age, years, mean (SD)	54.8 (13.6)	51.6 (15.6)	55.1 (13.4)	53.1 (15.2)	56.4 (13.1)	56.1 (14.7)	0.0001
Sex, no. (%)							
Female	6702	731 (10.9)	3263	464 (14.2) 14.22	643	110 (17.1) 17.11	<0.0001
Male	5131	1023 (20.0) 19.94	2440	573 (23.5) 23.48	509	119 (23.4) 23.38	0.0003
Race/ethnicity, no. (%)							
White	8464	1269 (15.0)	3895	738 (19.0)	809	161 (19.9)	<0.0001
Hispanic	1441	218 (15.1)	747	152 (20.4)	131	32 (24.0)	<0.0001
Black	1301	143 (11.0)	654	83 (12.7)	137	21 (15.3)	0.04
Asian	311	45 (14.5)	158	23 (14.6)	39	8 (19.4)	0.23
Other	316	79 (25.0)	249	41(16.5)	36	7 (20.5)	0.02
US residence, no. (%)	11,480	1675 (14.6)	5499	997 (18.1)	1111	224 (20.0)	<0.0001
HBV risk factor, no. (%)	3412	572 (16.8)	1668	356 (21.3)	311	88 (28.3)	<0.0001
Cancer type, no. (%)							<0.0001
Solid tumor^f^	9521	326 (3.4)	4602	208 (4.5)	908	47 (5.2)	<0.0001
Hematologic malignancy	2312	1428 (61.8)	1101	829 (75.3)	244	182 (74.6)	<0.0001
Chemotherapy							
Type, n (%)							
Rituximab	1244	785 (63.1)	606	481 (79.4)	127	94 (74.0)	<0.0001
Non-rituximab	10,589	969 (9.4)	5097	556 (10.9)	1025	135 (13.2)	<0.0001

*Abbreviations:HBV* hepatitis B virus, *SD* standard deviation, *US* United States.

^a^HBV screening means that both hepatitis B surface antigen (HBsAg) test and antibody to hepatitis B core antigen (anti-HBc) test were ordered.

^b^First chemotherapy administration from 1/1/04 through 12/18/2008.

^c^First chemotherapy administration from 12/19/2008 through 9/30/2010.

^d^First chemotherapy administration from 10/1/2010 through 4/30/11.

^e^Cochran-Armitage trend test compares screened patients vs. unscreened patients, over the 3 time periods.

^f^Excludes primary liver cancer.

Screening was almost always performed with both HBsAg and anti-HBc. Rates of use of the HBsAg test alone were 0.8% in period 1, 0.4% in period 2, and 0.9% in period 3 (*P* = 0.06). Among the 3020 screened patients, 252 (8.3%) had a positive result for either HBsAg or anti-HBc test. Specifically, 31 (1.0%) had positive results on both HBsAg and anti-HBc tests, 218 (7.2%) had a negative HBsAg test and a positive anti-HBc test, and 3 (0.1%) had a positive HBsAg but negative anti-HBc. Assuming that unscreened patients had negative tests, the proportions of patients with a positive result on either HBsAg or anti-HBc testing among all patients who received chemotherapy in periods 1, 2, and 3 were 1.4% (169/11,833), 1.5% (84/5703), and 1.7% (19/1152), respectively (*P* < 0.0001).

### Solid tumors

Among patients with solid tumors, screening rates for periods 1, 2, and 3, respectively, were as follows: breast: 2.1%, 2.2%, 5.8% (*P* = 0.01); lung: 1.1%, 2.9%, 2.9% (*P* = 0.009); colon: 3.5%, 4.6%, 3.4% (*P* = 0.30); and prostate: 2.8%, 2.9%, 2.8% *(P* = 0.37). The odds of HBV screening were increased by 30% and 70% for patients who had chemotherapy in periods 2 and 3, respectively, compared to period 1 (Table 4). Other significant predictors of higher rate of HBV screening were younger age, male gender, US residence, having at least 1 HBV risk factor, and planned rituximab therapy. HBV screening was performed in 64.4% of patients with and in 3.2% without rituximab in their chemotherapy regimen.

**Table 4:** **Predictors of HBV screening**^**a **^**by cancer type**

**Predictor**	**Hematologic malignancy (N = 3657)**					**Solid tumor**^**b **^**(N =15,031)**				
	**Screened**	**Univariate logistic regression**		**Multiple logistic regression OR**		**Screened**	**Univariate logistic regression**		**Multiple logistic regression**	
	**(N=2439) (66.7%)**	**OR (95% CI)**	***P *** **value**	**(95% CI)**	***P *** **value**	**(N=581) (3.9%)**	**OR (95% CI)**	***P *** **value**	**OR (95% CI)**	***P *** **value**
Age, years, mean (SD)	52.5 (15.5)	0.99 (0.99–1.0)	0.005	0.99 (0.98–0.99)	0.0001	52.4 (15.0)	0.98 (0.98–0.99)	<0.0001	0.98 (0.97–0.98)	<0.0001
Sex, no. (%)										
Male	1418/2133 (66.5)	Ref.	-	-	-	297/5947 (5.0)	Ref.	-	Ref.	-
Female	1021/1524 (67.0)	1.0 (0.89–1.2)	0.74	-	-	284/9084 (3.1)	0.61 (0.52–0.73)	<0.0001	0.58 (0.49–0.70)	<0.0001
Race/ethnicity, no. (%)										
White	1776/2645 (67.2)	Ref.	-	Ref.	-	392/10,523 (3.7)	Ref.	-	-	-
Hispanic	324/486 (66.7)	0.98 (0.80–1.2)	0.84	0.92 (0.75–1.1)	0.45	78/1833 (4.3)	1.1 (0.90–1.5)	0.27	-	-
Black	196/333 (58.9)	0.70 (0.56–0.88)	0.003	0.69 (0.55–0.88)	0.002	51/1759 (2.9)	0.77 (0.57–1.0)	0.09	-	-
Asian	41/50 (82.0)	2.2 (1.1–4.6)	0.03	2.0 (0.98–4.3)	0.06	35/458 (7.6)	2.1 (1.5–3.1)	<0.0001	-	-
Other	102/143 (71.3)	1.2 (0.8–1.8)	0.23	1.0 (0.72–1.6)	0.79	25/458 (5.5)	1.5 (0.98–2.3)	0.06	-	-
Residence, no. (%)										
US	2332/3510 (66.4)	Ref.	-	-	-	564/14,580 (3.9)	Ref.	-	Ref.	-
Outside US	107/147(72.8)	1.4 (0.93–2.0)	0.11	-	-	17/451 (3.8)	0.97 (0.59–1.6)	0.92	0.51 (0.30–0.90)	0.02
HBV risk factor, no. (%)										
No	1683/2603 (64.7)	Ref.	-	Ref.	-	321/10,694 (3.0)	Ref.	-	Ref.	
Yes	756/1054 (71.7)	1.4 (1.2–1.6)	<0.0001	1.3 (1.1–1.5)	0.001	260/4337 (6.0)	2.1 (1.7–2.4)	<0.0001	2.5 (2.1–3.0)	<0.0001
Chemotherapy type, no. (%)										
Non-rituximab	1191/1854 (64.2)	Ref.	-	Ref.	-	469/14,857 (3.2)	Ref.	-	Ref.	-
Rituximab	1248/1803 (69.2)	1.2 (1.1–1.4)	0.001	1.3 (1.2–1.5)	<0.0001	112/174 (64.4)	55.4 (40.1–76.6)	<0.0001	62.0 (44.1–87.0)	<0.0001
Timing of first chemotherapy^c^										
Period 1	1428/2312 (61.8)	Ref.	-	Ref.	-	326/9521 (3.4)	Ref.	-	Ref.	-
Period 2	829/1101 (75.3)	1.9 (1.6–2.2)	<0.0001	2.0 (1.6–2.3)	<0.0001	208/4602 (4.5)	1.3 (1.1–1.6)	0.001	1.3 (1.1–1.6)	0.003
Period 3	182/244 (74.6)	1.8 (1.4–2.4)	<0.0001	1.9 (1.4–2.6)	<0.0001	47/908 (5.2)	1.5 (1.1–2. 1)	0.007	1.7 (1.2–2.3)	0.003

*Abbreviations*: *HBV* hepatitis B virus, *OR* odds ratio, *CI* confidence interval, *Ref*., reference.

^a^HBV screening means that both hepatitis B surface antigen (HBsAg) test and antibody to hepatitis B core antigen (anti-HBc) test were ordered.

^b^Excludes patients with primary liver cancer.

^c^Period 1: 1/1/04 through 12/18/2008; period 2, 12/19/2008 through 9/30/2010; period 3, 10/1/2010 through 4/30/11.

### Hematologic malignancies

Among patients with hematologic malignancies, the screening rate increased during period 1 by 1% per quarter and then stabilized for periods 2 and 3 (Figure 2). This pattern was seen in lymphoma patients (63.5%, 81.3%, 81.3% for periods 1, 2, and 3, respectively; *P* ≤ 0.001) and acute leukemia patients (75.2%, 88.9%, 89.1% for periods 1, 2, and 3, respectively; *P* ≤ 0.001). The odds of screening were nearly twice as high for patients who had chemotherapy in period 2 as for patients who had chemotherapy in period 1 (Table 4). No incremental effect was observed after publication of national recommendations. Other significant predictors of screening were younger age, having at least 1 HBV risk factor, and planned rituximab therapy. HBV screening was performed in 69.2% of patients with and 64.2% of patients without rituximab in their chemotherapy regimen. Black race was associated with a lower screening rate.

**Figure 2:** **Trends in HBV Screening at MD Anderson Cancer, 2004–2011, in relation to publication of recommendations.** HBV screening prevalence is shown for patients with hematologic malignancies (blue line) and solid tumors (green line). Data points indicate average screening prevalence per quarter (Q) of each year. Q1, Jan 1-Mar 31; Q2, Apr 1-Jun 30; Q3, Jul 1-Sept 30; Q4, Oct 1-Dec 31. Numbers at top of figure refer to publication of national recommendations and associated reference number, as follows: 1, US Food and Drug Administration; 2, American Association for the Study of Liver Diseases (2007); 3, Centers for Disease Control and Prevention; 4, American Association for the Study of Liver Diseases (2009); 5, National Comprehensive Cancer Network; 6, Institute of Medicine; and 7, American Society of Clinical Oncology.

## Discussion

We found that the HBV screening prevalence among new patients receiving chemotherapy at a large US cancer center over the period 2004–2011 was only 16.2%. Of particular concern, the prevalence of HBV screening was low (<19%) even for patients with known HBV risk factors. Over 66% of patients with hematologic malignancies but less than 4% of those with solid tumors were screened. Predictors of HBV screening included having an HBV risk factor and planned rituximab therapy. Interestingly, race/ethnicity was associated with the likelihood of HBV screening for patients with hematologic malignancies but not with solid tumors. Importantly, HBV screening prevalence increased over time and higher rates were sustained after publication of national HBV screening recommendations. In this study of provider-driven screening, 8.3% of screened patients had a positive HBsAg or anti-HBc test result. The proportion of patients who tested positive for HBV infection increased by over 20% from period 1 to period 3, suggesting that increased screening may lead to increased identification of patients with HBV infection.

The finding that most patients with hematologic malignancies were screened for HBV infection whereas most patients with known HBV risk factors were not, together with the finding that most patients who received rituximab, a known risk factor for reactivation, were screened, suggests that oncologists are more aware of the risk factors for HBV reactivation than they are of the risk factors for HBV infection. This may have reflected the effect of the FDA letters, package inserts, and recommendations as well as publications in the oncology literature about HBV reactivation associated with rituximab treatment. These data indicate that future educational efforts on risk factors for HBV infection for oncology providers might increase HBV screening.

For patients with hematologic malignancies, the prevalence of HBV screening increased dramatically during period 1, which included the FDA letter. This increase may be related to the high risk (nearly 50%) of reactivation [16] and frequent reports of reactivation among patients with hematologic malignancies [17-19] and to the frequent reports of reactivation among patients receiving rituximab [20-24]. The further increase in screening prevalence during periods 2 and 3 was likely due to the emphasis in national recommendations on the risk of HBV reactivation in these patients.

For patients with solid tumors, odds of screening increased over all 3 time periods; however, the vast majority (96%) of patients were not screened. The low rate of HBV screening among patients with solid tumors is concerning because of previous reports of reactivation and related delays in chemotherapy and increases in mortality in patients with breast cancer [25-27], glioblastoma [28], germ cell tumors [27], and cancers of the lung, colon, and stomach [27,29-31]. Indeed, the risk of reactivation among patients with solid tumors is estimated to be approximately 15% [27]; however, these data were derived in an HBV-endemic area. Therefore, studies are needed to define risks and to determine predictors of reactivation for US patients with solid tumors.

Most of the national recommendations [1,2,4-7] call for prechemotherapy HBV screening in patients with high risk of HBV infection. Although the overall screening prevalence among patients with HBV risk factors was low, the prevalence increased over time, and having an HBV risk factor predicted screening. However, since previous studies have shown that screening based on risk factors alone would miss up to 45% to 65% of patients who actually had HBV infection, [32,33] future research is warranted to better understand the efficacy of risk-based screening.

Our study’s screening rate is lower than that in previous studies, which have described rates of adherence to cancer-related guidelines ranging from 27% to 97%, [34-41] although it is possible that our screening rates may have underestimated the actual rate since we could not verify HBV screening performed before registration at MD Anderson. Reasons for noncompliance with HBV screening guidelines may have included patient characteristics such as age [34,38] and stage of disease [34], physician attitudes towards guidelines [42], and education about guidelines [43]. One study [44] found that physicians’ lack of awareness of and lack of agreement with guidelines were potential barriers to adherence. A previous study by In et al. [45] reported a higher variation in surgical cancer care when guidelines were based on low levels of evidence or expert opinion. Future research providing high levels of evidence will be necessary to improve adherence to HBV screening.

We found that rituximab was a predictor of screening for all patients, especially those with solid tumors. Rituximab is a monoclonal antibody against CD20+ that causes severe B-cell depletion [46,47] and facilitates uncontrolled replication of HBV. However, besides rituximab, many other chemotherapy drugs [25-28,48-54] have been associated with HBV reactivation. Future studies focusing on mechanisms by which certain chemotherapy drugs may cause reactivation will help shape future evidence-based screening strategies.

Interestingly, whereas race/ethnicity did not predict HBV screening among patients with solid tumors, among patients with hematologic malignancies, Black patients had lower odds of screening than White patients. This is concerning because previous population-based studies have shown that the prevalence of HBV infection (current and past) is higher among Black than White adults (9.6% vs. 2.3%, *P* < 0.001) [55]. Perhaps physicians are unaware of the higher HBV risk in Black patients. We were surprised that Asian race did not predict HBV screening even though the prevalence of chronic HBV infection in this group may be as high as 20% [55-57]. Failure to screen Asian patients may have reflected lack of awareness by physicians of HBV risk factors [58,59]. In addition, we were surprised that patients with solid tumors who resided outside the US had lower odds of HBV screening, although it is possible that they were screened in their home countries.

We found substantial numbers of patients who had a negative HBsAg test result but a positive anti-HBc test result. Such patients may have occult HBV infection, as underscored by the high risk (78%) of HBV transmission in recipients transplanted with livers from donors with isolated anti-HBc positivity as compared to donors who were anti-HBc negative (0.05%) [60]. It is possible that isolated anti-HBc may represent false-positive test result among populations with a low prevalence of HBV infection. However, reactivation has been reported in patients who are HBsAg negative but anti-HBc positive during chemotherapy particularly if the regimen includes rituximab [21,24,61]. The ASCO PCO [7] recommends anti-HBc testing in some populations—e.g., patients with hematologic malignancies—since the risk of reactivation has been reported to be 10% among patients with hematologic malignancies with isolated anti-HBc [62]. The CDC recommends HBV screening using 3 HBV serology tests. We found that anti-HBs was rarely tested during our study period.

The strengths of our study include the large and heterogeneous patient population and the focus on actual rather than recalled HBV screening practice. Previous survey studies estimated 38%-80% of physicians screen patients before chemotherapy [11-13]; however, those results may inaccurately describe screening patterns since surveys record self-reporting of screening practice and not actual screening of individual patients. Our examination of physicians’ actual screening behavior at the level of individual patients avoided recall bias or subconscious attempts to report what should be done rather than what was actually done.

The main limitation of our study is its retrospective design and use of administrative databases, which prevented us from fully assessing HBV history and HBV risk factors. Patients may have received chemotherapy before their first chemotherapy administration at MD Anderson. Also, we excluded oral chemotherapy because we could not accurately access dispensing records outside of MD Anderson, but some oral chemotherapy could cause HBV. Patients’ race/ethnicity was self-described or assigned by referring clinics and may be incorrect. Another limitation is that we were not able to accurately determine prevalence of reactivation since not all patients who received chemotherapy were screened for HBV infection. This single-institution experience may not be generalizable to other settings, and our data cannot be generalized to patients who receive care in clinical trials as such patients were excluded. We did not explore socioeconomic factors such as income and educational level because this information is not part of our institutional Tumor Registry database. Most of our patients at MD Anderson have health insurance, and these plans are expected to pay for HBV screening tests. Finally, the last time period in our study was relatively short, limiting our ability to assess the full impact of the national recommendations. Nevertheless, our study provides valuable data from a large US academic cancer center with no changes in institutional policies regarding HBV screening during the study period.

## Conclusions

In conclusion, we found that the prevalence of HBV screening before chemotherapy among new patients receiving chemotherapy at a large US cancer center during 2004–2011 was only 16.2% overall but increased over time. The vast majority of patients with solid tumors, even those with risk factors for HBV infection, remained unscreened. Future research is needed to explore risks and predictors of reactivation with chemotherapy for US patients to develop evidence-based screening guidelines. Once these are available, educational efforts should be developed to increase oncology medical providers’ awareness of the importance of HBV screening and prophylaxis to prevent reactivation due to chemotherapy.

## Competing interests

The authors declare that they have no competing interests.

## Authors’ contributions

All authors contributed to the interpretation of data, to the critical revision of the manuscript for important intellectual content, and to the administrative, technical, and material support for this project. JPH was responsible for the conception and design of the study, acquisition of the data, and analysis and interpretation of data, drafting of the manuscript, and funding for the project. HZ performed the statistical analysis. MES-A contributed to the conception and design of the study as well as provided funding and supervision for the project. All authors read and approved the final manuscript.

## Pre-publication history

The pre-publication history for this paper can be accessed here:

http://www.biomedcentral.com/1471-2407/13/534/prepub
